The article "Antibacterial and Antioxidant Effects of Magnesium Alloy on Titanium Dental Implants" was retracted in 2023. Reasons: signs of a paper mill; compromised peer review; unreliable results or conclusions.

# Antibacterial and Antioxidant Effects of Magnesium Alloy on Titanium Dental Implants

**DOI:** 10.1155/2022/6537676

**Published:** 2022-01-06

**Authors:** Yang Bai, Lin Wang, Lisheng Zhao, E. Lingling, Shuo Yang, Shunyi Jia, Ning Wen

**Affiliations:** Department of Stomatology, The First Medical Center, Chinese PLA General Hospital, Beijing 100853, China

## Abstract

**Objectives:**

In this study, a new type of dental implant by covering the surface of the titanium (Ti) implant with zinc-magnesium (Zn-Mg) alloy was designed, to study the antibacterial and antioxidant effects of Mg alloy on titanium (Ti) implants in oral implant restoration.

**Methods:**

Human gingival fibroblasts (HGFs), S. sanguinis, and F. nucleatum bacteria were used to detect the bioactivity and antibacterial properties of Mg alloy-coated Ti implants. In addition, B6/J mice implanted with different materials were used to further detect their antibacterial and antioxidant properties.

**Results:**

The results showed that Mg alloy could better promote the adhesion and proliferation and improve the alkaline phosphatase (ALP) activity of HGFs, which contributed to better improved stability of implant osseointegration. In addition, Mg alloy could better inhibit the proliferation of S. sanguinis, while no significant difference was found in the proliferation of F. nucleatum between the two implants. In the mouse model, the peripheral inflammatory reaction and oxidative stress of the Mg alloy implant were significantly lower than those of the Ti alloy implant.

**Conclusions:**

Zn-Mg alloy-coated Ti implants could better inhibit the growth of Gram-positive bacteria in the oral cavity, inhibit oxidative stress, and facilitate the proliferation activity of HGFs and the potential of osteoblast differentiation, thus, better increasing the stability of implant osseointegration.

## 1. Introduction

In the daily diagnosis and treatment of stomatology, implants will be used in the process of repairing dentition defects to provide a solid base for the restoration of posterior crowns [1, 2]. However, there is also a probability of implantation failure, such as poor bone healing around the implant and inflammatory hyperplasia [3, 4], which will increase the risk of dental implant failure, cause adverse physical and mental effects to patients, and increase the medical burden. At present, titanium (Ti) is widely used in prosthodontics in virtue of its excellent mechanical strength and good biocompatibility [5]. However, due to the lack of antibacterial activity on the surface of pure Ti implants, implant placement creates a favorable environment for the growth and invasion of various positive and negative bacteria in the oral cavity, increasing the risk of infection. In addition, because of the lack of biological activity of pure Ti implant, their contact with alveolar bone can easily lead to slow healing with the surrounding bone and the acceleration of marginal bone loss, resulting in implant loosening [6]. Therefore, modifying the surface of Ti implants to improve their antibacterial activity and promote the attachment of bone cells is of great significance to improve the implant success rate [7].

The article "Antibacterial and Antioxidant Effects of Magnesium Alloy on Titanium Dental Implants" was retracted in 2023. Reasons: signs of a paper mill; compromised peer review; unreliable results or conclusions.

Preventing bone loss around dental implants, promoting bone healing, and maintaining osseointegration stability are important factors to ensure the success of dental implants. As an important ion in the process of bone healing, magnesium (Mg) is an essential nutrient element for the human body [8] and can be metabolized through kidney, with good biodegradability in vivo. With the increase of Mg concentration around the implant, the bone induction function is enhanced to promote the proliferation and differentiation of bone marrow mesenchymal stem cells, thus, playing an important role in the adhesion of the implant to the surrounding bone [9]. At the same time, Mg can prevent local hypercalcemia and hyperphosphatemia by regulating serum calcium and phosphorus levels, thus, avoiding local mineralization and better promoting bone healing [10]. Zinc (Zn), on the other hand, as an important microelement in bone metabolism, helps maintain the osseointegration stability after implant placement [11].

Oxidative stress is an important cause of inflammation. Therefore, inhibiting the production of reactive oxygen species (ROS) after implant placement is an important measure to reduce the release of inflammatory factors, thus, reducing body damage. Mg and Zn can regulate L-type calcium (Ca) channels in the body and reduce intracellular Ca concentration [12, 13], thus, avoiding the activation of intracellular Ca-dependent pathways. For example, the activation of nicotinamide adenine dinucleotide phosphate oxidase, which is the key enzyme of redox signal, will lead to a large number of ROS generation [14]. In addition, the activation of nitric oxide synthase will induce massive production of nitric oxide (NO) in vivo, thus, leading to the accumulation of peroxynitrite anion, a powerful oxidant in the body that cannot be effectively eliminated at present. Therefore, the activation of the above enzymes will significantly promote the occurrence of oxidative stress reaction in vivo, leading to inflammatory reaction. Mg has the function of regulating and inhibiting lipid peroxidation in vivo. Kostellow and Morrill [15] found that when the iron concentration was too high in vivo, it would lead to lipid peroxidation in the aortic root of mice. While local enrichment of high concentration of Mg can significantly inhibit the occurrence of iron catalyzed lipid peroxidation, thus, avoiding further damage to the fluidity and permeability of cell membrane and protecting the function and structure of cells. Moreover, by regulating the levels of Ca and phosphorus in vivo, Mg can avoid the stimulation of hyperphosphatemia and hypocalcemia on serum parathyroid hormone, thus, avoiding the release of inflammatory markers such as IL-6 [16]. In terms of antibacterial action, previous studies have shown that Zn can effectively inhibit Staphylococcus aureus and Escherichia coli [17]. However, there are few reports on the research of Zn-Mg alloy-coated Ti implants. Accordingly, this study discussed the antibacterial and antioxidant effects of Zn-Mg alloy-coated Ti implants and the improvement on osseointegration stability, which is of great significance to improve the success rate of implantation and reduce patients' healing time.

The article "Antibacterial and Antioxidant Effects of Magnesium Alloy on Titanium Dental Implants" was retracted in 2023. Reasons: signs of a paper mill; compromised peer review; unreliable results or conclusions.

## 2. Materials and Methods

### 2.1. Preparation of Mg Alloy-Coated Titanium Implants

A pure titanium plate with a size of 10 × 10 × 1 mm was prepared. And a chemical solution was prepared, in which HF and HNO3 were dissolved in H2O in a ratio of 1 : 4 : 5. The titanium plate was etched 3 times with the above solution for 5 minutes each time and then repeatedly cleaned with ultrapure water. After sufficient drying, Mg/Zn was coinjected into the treated titanium plate and deposited at 85°C for 1 h. Mg alloy was then coated on the surface of titanium plate using 3 V direct current (Figure 1).

### 2.2. Cell Culture and Grouping

Human gingival fibroblasts (HGFs) (CL-0356, Procell, Wuhan, China) were used to assess the cytocompatibility of Mg alloy modified Ti. The cells were cultured in 24-well plates for 24 h with Dulbecco Minimum Essential Medium (DMEM, 90%, BNCC351841, Bnbio, Beijing, China) containing 10% Fetal Bovine Serum (FBS, BNCC253589, Bnbio) in a cell incubator (51032124, Thermo Fisher Scientific, MA, USA) under the growth conditions of 37°C and 5% CO_2_ in air. Then, these cells were collected and diluted with phosphate-buffered saline (PBS) solution to 1 × 10^4^ cells/mL. After sterilization in the medical pressure cooker, Mg and Ti alloys were added to the bottom of the 12-well plate, respectively, and then 1 mL of the above cultured cell liquid was added to cover the metal surface. Subsequently, 2 mL 90% DEME together with 10% FBS was added into the culture plates, and the cells were divided into Mg alloy-Ti group and Ti group. Cell proliferation assay was performed by immunofluorescence with the anti-ki67 antibody (ab15580, Abcam, USA). The Goat anti-Rabbit IgG (H&L) (488&546) was used as second antibody, and labeled cells were analyzed under flourescence microscopy.

The article "Antibacterial and Antioxidant Effects of Magnesium Alloy on Titanium Dental Implants" was retracted in 2023. Reasons: signs of a paper mill; compromised peer review; unreliable results or conclusions.

### 2.3. Bacteria Culture and Live/Dead Test

S. sanguinis (ATCC49295, Huzheng, Shanghai, China) and F. nucleatum (XYSW-JZ-2903, Xuanya, Shanghai, China), which represent the common gram-positive and gram-negative bacteria in the oral cavity, were used to detect the bacterial growth in Ti- and Mg-alloy. S. sanguinis strains were cultured in a 24-well plate for 24 h with glucose broth (LA3850, Solarbio, Beijing, China) in a microorganism incubator (51028133, Thermo Fisher Scientific) under 37°C with 5% CO_2_ in air. The colony inoculation concentration was adjusted to 108 CFU/mL, and Mg and Ti alloys were added to the bottom of the 12-well plate, respectively, after sterilization in the medical pressure cooker. Then, 1 mL S. sanguinis suspension and 2 mL glucose broth were added into culture plates and then cultured in the above culture environment for another 4 h in the dark. F. nucleatum strains were cultured in a 24-well plate for 24 h with ATCC® Medium 260 (Trypticase soy agar, brother, defibrinated sheep blood) in a microorganism incubator under 80% N2, 10% H_2_, and 10% CO_2_. The growth of F. nucleatum in Ti- and Mg-alloy was detected by the same method as S. sanguinis. The activation of S. sanguinis and F. nucleatum was tested by live/dead bacterial viability kit (04511, Sigma-Aldrich, St. Louis, MO, USA). In this kit, calcein AM solution was applied to live bacteria staining, which would release green fluorescence. For dead bacteria, they are stained with propidium iodide solution to release red fluorescence.

### 2.4. Detection of Alkaline Phosphatase (ALP) Activity in Cultured HGFs

The HGFs of Ti and Mg alloy-Ti group were cultured for 24 h and washed with PBS solution for 3 times after the removal of the original culture medium. Then, 200 *μ*L cell lysis reagent (C2360, Sigma-Aldrich) was added to the cells for digestion, after which the lysed cell liquid was placed in the ALP detection board to detect ALP activity. The detection process was strictly according to the detection method of alkaline phosphatase kit, and ALP activity was detected at 520 nm wavelength. In addition, the PBS solution was used as blank control.

### 2.5. Implant Surgery in Animals

Sixteen 12-week-old male B/6J mice with an average weight of about 250 g were purchased from Saiye (Suzhou) Biotechnology Co., Ltd. They were selected as experimental subjects to test the inflammatory response and oxidative stress response induced by implants in vivo. This study was approved by the Animal Ethics Committee of PLA General Hospital and the whole experiment followed all government regulations on the ethical use of animals. After general anesthesia with 10% chloride hydrate (0.4 mL/100 g), the implant was implanted in the central area of the mouse's back. A 2 cm long incision was made at 1 cm of the horizontal line of the scapula to expose the bone. After implantation, the muscle tissue and skin of mouse back were sutured intermittently.

The article "Antibacterial and Antioxidant Effects of Magnesium Alloy on Titanium Dental Implants" was retracted in 2023. Reasons: signs of a paper mill; compromised peer review; unreliable results or conclusions.

### 2.6. Antioxidation Test in the Mouse Model

Three weeks later, venous blood was collected from the mouse posterior orbital venous plexus and stored at -80°C in a medical refrigerator. In this study, superoxide dismutase (SOD), malondialdehyde (MDA), and total antioxidant capacity (TAC) were used to evaluate the degree of oxidative stress of implants in vivo. Mouse venous blood samples were obtained and centrifugal at 3000 r/min, and the supernatant was collected for the detection of oxidative stress. Superoxide Dismutase Activity Assay Kit (ab65354, Abcam) was used to test SOD, MDA was tested by ELISA Assay Kit (LE-M2471, Hefei Laier Biotechnology Co., Ltd), and TAC was detected by the fluorescence recovery after photobleaching (FRAP) method with Total Antioxidant Capacity Assay Kit (S0116, Beyotime, Shanghai, China).

### 2.7. Detection of Inflammatory Factors in Mouse

The venous blood samples of mice in each group were taken out from the medical refrigerator and centrifuged at 3000 r/min. The resulting supernatant was collected to test the levels of IL-6, IL-1*β*, and TNF-*α* using the mouse IL-6 ELISA Kit (ab222503, Abcam), mouse IL-1*β* ELISA Kit (ab197742, Abcam), and mouse TNF-*α* ELISA Kit (ab208348, Abcam), respectively.

### 2.8. Foreign Body Reaction Observation

Hematoxylin-eosin (HE) staining was used for foreign body reaction detection after implant placement. After the mice were sacrificed, the tissue around the implant was sampled, embedded in paraffin, and stained with HE. Local fiber growth pattern and immune cell infiltration were observed under microscopy.

### 2.9. Statistical Processing

SPSS22.0 statistical software and Graphpad Prism 6.0 were used for statistical analysis and visualization of the data, respectively. Mean ± standard deviation (mean ± SD) was used to describe quantitative data; the difference between groups was identified by independent samples *t*-test, with *P* < 0.05 as the significance level and 95% as the confidence interval (CI).

## 3. Results

### 3.1. Bioactivity Evaluation of Ti and Mg Alloy Implants In Vitro

As the most abundant cells in gingival connective tissue, the activity of HGFs plays a decisive role in maintaining the integrity and biological function of periodontal tissue. In this study, it was found that compared with Ti alloy and Mg alloy could better increase the adhesion and proliferation activity of HGFs to repair the periodontal tissue around the implant better (Figures 2(a)–2(d)). Under certain conditions, HGFs have the potential to differentiate into osteoblasts, which can repair the alveolar bone around the implant and further increase its stability. The activity of osteoblasts can be reflected by ALP. The experimental results showed that the ALP level of HGFs in Mg alloy-Ti group was higher, suggesting that Mg alloy could better induce the osteogenic ability of HGFs, thus, increasing the stability of implant osseointegration (Figure 2(e)).

The article "Antibacterial and Antioxidant Effects of Magnesium Alloy on Titanium Dental Implants" was retracted in 2023. Reasons: signs of a paper mill; compromised peer review; unreliable results or conclusions.

### 3.2. Bacteriostatic Evaluation of Ti and Mg Alloy Implants In Vitro

Due to food residues, oral bacteria are easy to breed. After implant placement, the gap between implant and soft tissue interface is prone to bacterial infection, which will lead to periodontal tissue destruction, affecting the stability of the implant. In this study, S. sanguinis and F. nucleatum were selected to represent Gram-positive and Gram-negative bacteria in oral cavity, respectively, so as to evaluate the antibacterial efficacy of Mg alloy and Ti alloy. The results showed that Mg alloy could better inhibit the proliferation of S. sanguinis (Figures 3(a) and 3(b)) and produce more dead bacteria (Figures 3(c) and 3(d)). In terms of F. nucleatum, both implants had no significant antibacterial effect on Gram-negative bacteria, so corresponding antibiotics should be used after implantation to avoid Gram-negative infection (Figures 3(e)–3(h)).

### 3.3. Histological Alteration around Implants In Vivo

Three weeks after implantation, we evaluated the foreign body reaction by HE staining. Obviously, there was less fibroblast reaction and inflammatory cell infiltration around the Mg alloy-coated Ti implant (Figures 4(a) and 4(b)), while there was more fibrous proliferation and chronic inflammatory cell infiltration around the Ti alloy implant (Figures 4(c) and 4(d)). Therefore, compared with Ti alloy, Mg alloy had better histocompatibility and less rejection.

### 3.4. Inflammation Response Caused by Implants In Vivo

Oral implants have high biocompatibility with the body, but as foreign bodies, they will cause foreign body reaction in vivo, leading to the aggravation of inflammation level. The inflammation level is closely related to implant success. This study found that the levels of inflammatory factors in Mg alloy-Ti group, including IL-1*β*, IL-6, and TNF-*α*, did not increase as much as those in Ti group after implantation (Figure 5). It was suggested that Mg alloy could better reduce the inflammatory reaction.

The article "Antibacterial and Antioxidant Effects of Magnesium Alloy on Titanium Dental Implants" was retracted in 2023. Reasons: signs of a paper mill; compromised peer review; unreliable results or conclusions.

### 3.5. Degree of Oxidative Stress Response Caused by Implants In Vivo

Oxidative stress is an important mechanism leading to inflammation. Therefore, detecting the degree of oxidative stress can effectively evaluate the inflammation degree after implantation. The results showed that compared with Ti group, the levels of SOD and TAC in Mg alloy-coated Ti group increased more significantly, and the level of MDA decreased more obviously (Figure 6). Therefore, Mg alloy had better antioxidative stress capacity.

## 4. Discussion

The oral cavity is where bacteria tend to accumulate. Relevant studies have shown that there are about 10000 bacterial phenotypes in the oral cavity [18]. So, once oral cavity is damaged, it is easy to be complicated with bacterial infection. Ti alloy is the most widely used metal implant in dental implant repair, which can provide a stable base for the later crown restoration [19]. However, after implant placement, bacteria in the oral cavity will invade through the gap between the implant and the periodontal tissue, causing inflammation and osseointegration instability, eventually resulting in the occurrence of implant failure [20]. Therefore, how to accelerate gap sealing and inhibit bacterial invasion has become a research hotspot to improve the implant success rate. Recently, it has been an important way to solve the above problems by modifying the implant surface, endowing implants with antibacterial properties, and improving the biological activity of the surrounding cells. Mg, as an important element in the body, is involved in bone healing and plays an anti-inflammatory and antioxidation role by regulating Ca channels [16, 21]. In addition, it can be excreted with urine and reabsorbed through renal tubules, with good biodegradability in vivo. Therefore, modifying the surface of Ti implants with Mg alloy is of great significance to improve the success rate of implant repair and prolong the service life of implants.

HGFs are the most important cells in gingival tissue, and its proliferation activity directly affects the regeneration and consequently the integrity and biological function of periodontal tissue [22, 23]. In addition, relevant studies have shown that under certain conditions, HGFs have the potential to differentiate into osteoblasts, which can repair alveolar bone [24]. Therefore, studying the changes of HGFs activity after implant placement is of great significance for predicting the success of implantation. In this study, it was found that the proliferation of HGFs was better in Mg alloy-Ti group. Zhang et al. [25] found that Mg alloy-coated Ti implants had good osteoconduction and can promote the proliferation of bone cells, thus, enhancing the bearing capacity of implants. After implant placement, the alveolar bone is absorbed at its edges due to stimulation, while to maintain the implant stability, the periodontal tissue will migrate upward to the implant neck to obtain good osseointegration. Therefore, the increased activity of HGFs can better promote its adhesion to the implant surface and make the connection between cells tighter, thus, promoting the periodontal tissue repair at the interface between the implant and the soft tissue [26]. Closure of this gap can not only reduce the invasion of oral bacteria but also increase the implant stability, thus, improving the success rate of implants. In addition, the ALP activity of Mg alloy-Ti group significantly increased. ALP is involved in bone formation and its activity can reflect the osteogenic ability of cells. The above result suggests that Mg alloy can better induce the osteogenic capability of HGFs, so as to repair the damaged alveolar bone and further increase the stability of implant osseointegration.

The article "Antibacterial and Antioxidant Effects of Magnesium Alloy on Titanium Dental Implants" was retracted in 2023. Reasons: signs of a paper mill; compromised peer review; unreliable results or conclusions.

The occurrence of inflammation around the implant will cause periodontal tissue destruction and alveolar bone absorption, which will affect the implant stability and ultimately lead to the implantation failure. Oxidative stress is an important mechanism leading to inflammation. Therefore, the oxidative stress response at the implant soft tissue interface must be suppressed to avoid the continuous accumulation of ROS, thereby inhibiting the occurrence of inflammatory cascade [27, 28]. In this study, we found that Mg alloy could significantly inhibit oxidative stress reaction and reduce the damage of periodontal tissue, thus, better promoting the recovery of periodontal tissue and maintaining the implant stability. In addition, it can reduce the release of inflammatory factors, further reducing the inflammatory reaction and avoiding alveolar bone absorption. Moreover, Mg alloy could better inhibit the proliferation of S. sanguinis and inhibit the invasion of oral bacteria around the implant, thereby preventing HGFs from releasing inflammatory factors after being stimulated by pathogenic bacteria, and better maintaining their physiological functions.

## 5. Conclusion

In this study, we investigated the antibacterial and antioxidant properties of Zn-Mg alloy-coated Ti implants. We found through in vitro experiments that Mg alloy could better maintain the activity of HGFs, thus, promoting periodontal tissue repair. In addition, it can induce HGFs to differentiate into osteocytes to promote the repair of alveolar bone and better maintain the stability of implants. Furthermore, Mg alloy could significantly inhibit the proliferation of S. sanguinis, which is conducive to reducing the inflammatory reaction and better maintaining the biological activity of HGFs. Moreover, Mg alloy has a good antioxidative stress effect and can inhibit the release of inflammatory factors. Therefore, Mg alloy implants, which can better inhibit the growth of Gram-positive bacteria in the oral cavity and increase the stability of implant osseointegration, can be used in dental implant restoration in the future, with great significance in improving the success rate of implantation and shortening the healing time of patients.

The article "Antibacterial and Antioxidant Effects of Magnesium Alloy on Titanium Dental Implants" was retracted in 2023. Reasons: signs of a paper mill; compromised peer review; unreliable results or conclusions.

## Figures and Tables

**Figure 1:** Schematic diagram of Mg alloy-coated Ti implant and its capacity of anti-inflammatory and antioxidation.

**Figure 2:** Effects of implants on the bioactivity of HGFs. (a) The growth pattern of HGFs on the surface of Ti implant. (b) The growth pattern of HGFs on the surface of Mg alloy-coated Ti implant. (c) Ki-67 expression of HGFs on the surface of Ti implant. (d) Ki-67 expression of HGFs on the surface of Mg alloy-coated Ti implant. (e) Quantitative evaluation of ALP relative activity in HGFs between Mg alloy-Ti and Ti group. Test method: Student's *t* test, ∗∗*P* < 0.01.

**Figure 3:** Growth of S. sanguinis and F. nucleatum on implant surface. (a) Live staining of cultured S. sanguinis bacteria 4 h after adding Ti implant. (b) Live staining of cultured S. sanguinis bacteria 4 h after adding Mg alloy-coated Ti implant. (c) Dead staining of cultured S. sanguinis bacteria 4 h after adding Ti implant. (d) Dead staining of cultured S. sanguinis bacteria 4 h after adding Mg alloy Ti-coated implant. (e) Live staining of cultured F. nucleatum bacteria 4 h after adding Ti implant. (f) Live staining of cultured F. nucleatum bacteria 4 h after adding Mg alloy Ti-coated implant. (g) Dead staining of cultured F. nucleatum bacteria 4 h after adding Ti implant. (h) Dead staining of cultured F. nucleatum bacteria 4 h after adding Mg alloy Ti-coated implant.

**Figure 4:** Histological appearance of surrounding tissue after implant placement in Mg alloy-Ti group ((a) and (b)) and Ti group ((c) and (d)).

**Figure 5:** Inflammatory evaluation of different implant materials. (a) Blood IL-1*β* level 3 weeks later in Mg alloy-Ti group and Ti group. (b) Blood IL-6 level 3 weeks later in Mg alloy-Ti group and Ti group. (c) Blood TNF-*α* level 3 weeks later in Mg alloy-Ti group and Ti group. Test method: Student's *t* test, ∗∗*P* < 0.01.

**Figure 6:** Comparison of antioxidation capacity between Mg alloy-Ti group and Ti group. (a) SOD concentration. (b) MDA concentration. (c) TAC concentration. Test method: Student's *t* test, ∗∗*P* < 0.01.

The article "Antibacterial and Antioxidant Effects of Magnesium Alloy on Titanium Dental Implants" was retracted in 2023. Reasons: signs of a paper mill; compromised peer review; unreliable results or conclusions.

## Data Availability

The labeled dataset used to support the findings of this study are available from the corresponding author upon request.
